# Association Mining of Near Misses in Hydropower Engineering Construction Based on Convolutional Neural Network Text Classification

**DOI:** 10.1155/2022/4851615

**Published:** 2022-01-03

**Authors:** Shu Chen, Junbo Xi, Yun Chen, Jinfan Zhao

**Affiliations:** ^1^Department of Engineering Management, College of Hydraulic and Environmental Engineering, China Three Gorges University, Yichang, Hubei 443002, China; ^2^Department of Engineering Management, College of Economics and Management, China Three Gorges University, Yichang, Hubei 443002, China

## Abstract

Accidents of various types in the construction of hydropower engineering projects occur frequently, which leads to significant numbers of casualties and economic losses. Identifying and eliminating near misses are a significant means of preventing accidents. Mining near-miss data can provide valuable information on how to mitigate and control hazards. However, most of the data generated in the construction of hydropower engineering projects are semi-structured text data without unified standard expression, so data association analysis is time-consuming and labor-intensive. Thus, an artificial intelligence (AI) automatic classification method based on a convolutional neural network (CNN) is adopted to obtain structured data on near-miss locations and near-miss types from safety records. The apriori algorithm is used to further mine the associations between “locations” and “types” by scanning structured data. The association results are visualized using a network diagram. A Sankey diagram is used to reveal the information flow of near-miss specific objects using the “location ⟶ type” strong association rule. The proposed method combines text classification, association rules, and the Sankey diagrams and provides a novel approach for mining semi-structured text. Moreover, the method is proven to be useful and efficient for exploring near-miss distribution laws in hydropower engineering construction to reduce the possibility of accidents and efficiently improve the safety level of hydropower engineering construction sites.

## 1. Introduction

Construction is a high-risk industry, and until recently, construction sites have continued to pose a serious threat to workers' lives and health [1]. In particular, hydropower engineering construction leads to various types of casualties due to the frequent cross-work of construction equipment, the dynamic construction work environment, and high-risk site operations [2]. For example, in March 2020 alone, there were two hydropower accidents in Sichuan Province: a scaffolding collapse and high falls caused by burnt-out safety belts led to 3 deaths and 4 injuries, according to China's National Energy Administration [3].

Near misses have been defined as a dangerous state in production that may lead to accidents, such as the unsafe behavior of people, an unsafe state of things, unsafe factors in the environment, and defects in management [4]. In particular, there is a wider variety of near misses in the construction of hydropower engineering, leading to a sharply increased probability of serious accidents. An accident is a fait accompli and cannot be undone. In contrast, near misses still have remedial leeway [5]. Therefore, to improve the safety situation, it is a key part of safety management to determine the potential laws of near misses and take safety measures to eliminate near misses in the construction of hydropower engineering projects.

With increasing attention to safety issues in the hydropower industry, the frequency of safety inspections has increased rapidly, and numerous near-miss text data have been accumulated. However, text data are both semi-structured and unstructured; accordingly, traditional methods of mining text data are time-consuming and labor-intensive. With the development of artificial intelligence (AI) technology, automatic mining and analysis of near misses will inevitably replace relying on manual work to structure text data and find near-miss laws [6]. Thus, it is of great significance to study the data mining of near-miss text data, especially the mining of near-miss distribution laws relying on AI technology.

In the field of construction, text mining application research mainly adopts text classification methods to classify housing construction accidents, subway construction near misses, and construction contract documents. Shallow machine-learning algorithms, such as the support vector machine (SVM), naive Bayes (NB), and K-nearest neighbor (KNN) algorithms, have been used to classify housing construction accidents [7] and construction contract documents [8]. Such algorithms require manually combining lexical, syntactic, and semantic features. These are limited by the domain knowledge of individuals, resulting in poor performance in feature representation.

In contrast, deep learning algorithms (e.g., convolutional neural networks (CNNs) [9], Bidirectional Encoder Representations from Transformers (BERT) for language understanding [10], and convolutional bidirectional long short-term memory (C-BiLSTM) [11]) can automatically identify features and use existing tagged data to train the classification model of house-building construction accidents and near-miss subway construction. The above research proves that deep learning has a better effect on the classification of construction of short texts than shallow machine learning.

Previous text information expression and big data mining technology have laid a very important foundation for intelligent analysis of text information. All kinds of text intelligent analysis technology have been widely used in housing construction, subways, and so on. However, there are few studies on the intelligent analysis of big data in the field of safety knowledge in hydropower engineering construction addressed in this study. Although the core algorithm of text big data analysis has not changed much, due to the unique characteristics of safety knowledge in hydropower engineering construction, the data analysis framework that focuses on hidden trouble needs to be reformulated. The main reason is that hydropower engineering construction involves a wide range of engineering types, and there are huge differences between different engineering types, leading to the necessity of reexploring the distribution of near misses in this kind of engineering. Moreover, these studies only classified the text without discussing how to further mine the more detailed construction knowledge contained in the classified text. Safety managers cannot intuitively and quickly acquire near-miss knowledge due to the poor visualization effect of near-miss distributions.

Against this contextual backdrop, we develop a near-miss classifier based on a CNN, associate the classified results, and visualize them with a network diagram [12] and a Sankey diagram so that safety managers can easily find the key points of massive near misses [13]. First, to structure text data, a CNN-based classifier that incorporates a deep learning method is developed to generate structured classification results of near-miss information within safety records. The classifier can capture semantic features in a near-miss text to automatically classify near-miss locations and the near-miss descriptions into predefined “location” and “type” categories, which can generate structured data for statistical analysis. An apriori algorithm is then used to quantify the frequency and trustworthiness of the association rule “location ⟶ type.” The network diagram visualizes the quantification of the association rule “location ⟶ type.” Finally, after integrating all texts corresponding to each category of strong association rules, the Chinese word segmentation is carried out on these texts. A Sankey diagram is drawn with word frequency as the size of the information flow.

A classifier based on deep learning and a CNN combined with the apriori algorithm and a Sankey diagram can automatically classify text and associate the “location” and “type” of the classification results. Consequently, safety management personnel can implement corresponding near-miss measures for specific near-miss locations, eliminate near misses in advance, and improve the safety level of hydropower project construction.

## 2. Related Work

### 2.1. Accident Prevention in Hydropower Engineering Construction

Hydropower engineering construction has the characteristics of a complex construction environment, including a wide range of cross-work and high labor intensity. Moreover, it has a low level of safety management and, more generally, a lack of safety supervision and personnel training [14]. Accidents occur frequently in hydropower project construction. There are many studies on accident prevention in hydropower engineering construction. Zheng et al. [15] applied the Human Factor Analysis and Classification System (HFACS) to study the evaluation of human factors in high-risk operations and finally obtained the evaluation value of faulty behavior risk (FBR) in hydropower engineering construction. Zhou et al. [2] integrated the methods of the decision-making trial and evaluation laboratory (DEMATEL) and the analytic network process (ANP), taking into account the interaction between factors and their self-feedback. The deduced causal diagrams provide suggestions for the safety management of high-risk working systems in several large hydropower projects. Zheng et al. [16] adopted the HFACS framework, collected 869 accident investigation reports, determined the first three accident types by frequency statistics, and determined the accident path by analyzing the correlation between different human factors. All the above studies focus on the prevention of accidents, but the study of near misses can advance the link of accident prevention and reduce the probability of accidents by eliminating near misses.

### 2.2. Text Classification and Machine Learning

Natural language processing (NLP) is a technology in which a computer is used to process and analyze human language, including text classification, information extraction, and information retrieval [17]. Text classification is a common task of NLP, which concerns training mathematical models to gain a certain generalization ability by inputting a group of texts with relevant classification labels so that the model can better predict the categories of other texts in the same field [18]. Text classification has been widely used in various fields as an efficient information processing technology [19].

Machine learning is a popular method to realize text classification [20]. For instance, Bertke et al. [21] identified the three “claim cause” categories of workers' medical compensation claims using the NB classifier. Ubeynarayana et al. (Ubeynarayana. and Miang., 2017) used a support vector machine (SVM) classifier to classify the Occupational Safety and Health Accident (OSHA) dataset. Similarly, Mahfouz [8] utilized an SVM to classify unstructured information in contract documents. Maia et al. [22] used the random forest (RF) method to classify complaint texts and achieved good results. All of the above studies used shallow machine learning, which can only obtain simple functions through a linear combination of feature parameters of training data. However, simple functions poorly classify the complex and changeable near-miss text of hydropower project construction.

Deep learning (DL) can learn complex functions and extract higher-dimensional features from input data. The DL method has been identified as an appropriate method to automatically extract features for text classification without manually creating features [23]. Compared to shallow machine learning, DL can effectively extract word order features and learn from the semantic information contained in text [24].

CNNs have been applied in NLP and have achieved good results in semantic processing [25], sentence modeling [26], and search query retrieval [27]. Researchers are increasingly interested in the application of CNNs in text classification. Arora et al. [28] proposed a text normalization algorithm based on deep convolutional character level embedding (the Conv-char-EMB neural network model) for sentiment analysis (SA) of unstructured data. He et al. [29] proved that CNN architecture with multiple pooling operations can extract the most significant features of a convolutional filter by convolution, activation, and pooling operations and effectively classify medical relations.

Do [30] proposed a CNN model that can use both a word vector adjusted for a specific task and a static pretrained word vector for the sentence-level text classification task. Yoon et al. [31] used a CNN to classify sentences preprocessed by word embeddings and suggested that only one layer of convolution can classify sentences effectively. The above studies have laid an important foundation for text big data mining, but the laws contained in text big data of near misses in hydropower project construction need to be further explored. Due to the large difference in the characteristics of various subprojects for hydropower projects, the types of near misses in different locations are also very different and present great trouble in the analysis of hidden danger data. The text intelligence analysis method commonly used in other projects has difficulty addressing this challenge.

### 2.3. Association Rules and Sankey Diagram

Association rules contain the rules of occurrence between things. It is imperative for people to understand detailed information about the research object. Agrawal [32] proposed an association rule algorithm for mining the potential association between transactions in a transaction database. The apriori algorithm is the most famous association rule algorithm. It can prune item set trees to prevent the exponential growth of candidate item sets, reduce the amount of data, and improve operation efficiency [33].

Association rule mining has been widely used in construction safety fields. Cheng et al. [34] used association rules in analyzing 1347 accidents to identify potential hazards in Taiwanese construction projects. Guo et al. [35] found the association rules of workers' unsafe behavior, worker type, and construction phase in the construction industry using the apriori algorithm. Qiu and Wang [36] proposed the “cause ⟶ emergency measure” association rule algorithm based on construction accident cases to find all possible accident cause chains. Mingyuan et al. [37] used the apriori algorithm to mine a dataset of near misses in construction and obtained the correlation between the hazard sources in the internal and external environments of a construction site.

Using the apriori algorithm for data mining, these researchers obtained valuable association rules that are difficult to find by subjective experience. The algorithm involves counting the number of terms. For unstructured text, items that have the same meaning but different expressions are considered different when they are counted. Therefore, items with the same meaning need to be classified into the corresponding preset categories to obtain structured text. Finally, the number of items in each category is counted as the operation data of the apriori algorithm. However, the association rule algorithm is only applicable to mining structured data, it is necessary to carry out structured data tasks to mine unstructured text, and text classification plays such a role. Since the near misses of hydropower projects are recorded artificially, they are random and nonstandard, and all belong to unstructured texts. To mine the association rules of near misses of unstructured texts, it is necessary to obtain structured texts that are easy to calculate by classifying near misses.

A Sankey diagram is a data flow diagram that shows the flow of information among multiple attributes [38]. The Sankey diagram is a fashionable tool in energy system analysis [39], and it can clearly show the energy flow process. There are also some applications of the Sankey diagram in civil engineering. For example, Abdelalim et al. [40] used a Sankey chart to carry out data visualization and analysis of energy flow at the multizone building scale. Goswein et al. [41] used a Sankey diagram to represent the relationship between building stock and its driving factors. Ioannidou et al. [42] visualized the economic flow of construction projects through a Sankey diagram. These studies took advantage of the characteristic that the Sankey diagram can represent information flow. The distribution law of near misses also has the characteristics of information flow, so the Sankey diagram can be used to show the flow of specific near-miss objects between near-miss locations and near-miss types.

## 3. Data Preparation

The data preparation section is divided into 4 steps: (1) collecting near-miss data from the Crane Beach Hydropower Station projects and storing them in the database, (2) cleaning up noncompliance data and obtaining word segmentation, (3) labeling the training data, and (4) assigning the labeled dataset for training the model. This process is shown in Figure 1.

### 3.1. Source of Data

The 32,370 safety records of the Crane Beach Hydropower Station from 2015 to 2020 were taken as the data source. The 24,325 collected semi-structured records were uploaded by the site construction operator through WeChat-based near-miss check software. The 8045 paper unstructured records were collected from the safety management personnel at the construction site and manually entered into the database. Some examples of raw data are shown in Table 1.

Each near-miss record includes its check date, near-miss description, and near-miss location. In the near-miss records, “description” and “location” belong to semi-structured data, which are characterized by lengthy sentences and inconsistent expressions. The fields of a semi-structured record are related to each other, but the data stored in the fields are unstructured text. The “description” contains the information of the type of near misses, and the “locations” contain the information of the near-miss places. However, the information is unstructured text and cannot be associated with the association rule algorithm. To automatically find the association rules between the near-miss type and the near-miss location, these two fields need to be transformed into structured text. The CNN DL algorithm is used to transform these two fields into structured data, which are 11 near-miss types and 35 near-miss locations.

### 3.2. Data Preprocessing

The training effect of the model can be improved by preprocessing data to reduce data noise. The data preprocessing steps are as follows:

- Empty items, numbers, and punctuations such as “3#,” “/,” “,” and “6–2” in a sentence are considered noise, and regular expressions (REs) are used in Python to remove the noise. In particular, “3#” describes the location information of hydropower projects in a more specific way. In different # hidden trouble locations, the impact on hidden trouble types can be ignored, so 3# is not considered.
- Jieba [45] (Chinese word segmentation software based on Python) is employed to carry out word segmentation to better express the features of Chinese sentences.
- One-character words that are not rich in meaning are deleted.

### 3.3. Label Definition

Since a supervised learning model is proposed, it is necessary to label the classified data accurately. According to 20 accident types that a near miss may cause [44] and combined with the description of the near misses in this study, the near misses are divided into 11 types for hydropower engineering construction. Due to the differences in construction organization plans in each near-miss location, we define a total of 30 near-miss location labels. The text datasets are manually tagged by experienced safety management personnel on-site and then reviewed by experts in the field of hydropower engineering construction to ensure the accuracy of the labels. Partial labels are listed in Table 2.

### 3.4. Dataset Division

To obtain the classification model, the labeled datasets need to be divided into a training set, test set, and validation set. Among them, the training set optimizes the model, the validation set selects the parameters of the optimization model, and the test set evaluates the performance of the established model. The two datasets of “location” and “description” are arranged in proportion as follows: training set: test set: validation set = 10 : 1:1. The numbers of training sets, validation sets, and test sets for the “location” classifier are 14,995, 1515, and 1500, respectively. The numbers of training sets, verification sets, and test sets for the “type” classifier are 16,018, 1545, and 1580, respectively.

## 4. Near-Miss Text Mining Approach

The data mining model is divided into 3 parts: (1) CNN classification: the “type” classifier and “location” classifier are obtained by training the tag dataset. (2) Association analysis: the trained classifier classifies the “type” and “location” of new near misses to generate structured data of “type” and “location” for statistical analysis. An association rule network diagram is created to visualize the mining results. (3) Sankey diagram: the Sankey diagram adds detailed rules to the near-miss association rules. The specific steps are shown in Figure 2.

### 4.1. CNN-Based Classifier

The CNN is a supervised learning method in DL. The weight sharing of a convolutional layer in a CNN can reduce the number of trainable parameters in the network and the complexity of the network model. A text classification method based on CNN can learn complex functions and related features from a given text without the need to select effective features through tedious manual text analysis. This can greatly save on labor and time [9]. With the proposal of the word2vec method, word embedding training can be carried out on a large scale. This lays a foundation for CNN's extensive application in text classification [45].

The context information of each word in the near-miss text is crucial for the CNN model to capture the near-miss features. By introducing word2vec to the input layer, the near-miss text is transformed into a word embedded with a specific numeric expression containing the relationship between words in a near-miss text. This serves as the input layer of the CNN model. In the convolutional layer, the feature mapping of near-miss text is learned in parallel using different sizes of convolution kernels. A fixed-length near-miss feature mapping is acquired by performing the max pool operation at the pooling layer. The final near-miss classification task is handled by the full connection layer. This is equivalent to classifying the features extracted by the convolution layer and pooling. The model structure is shown in Figure 3.

#### 4.1.1. Word Representation

To make full use of the word characteristics, 19,143 “description” and 18,010 “location” instances in the dataset are divided into multiple words separated by line breaks with Jieba. Different words in the “description” and “location” datasets constitute the “description” word vector space and “location” word vector space, respectively. The numbers of words in the two word vector spaces are *V*_description_=8001 and *V*_location_=1919.

The text dataset of hydropower project construction near misses has the characteristics of a large word space, short sentences, and high frequency of professional vocabulary [46]. To better express the near-miss texts, we use word embedding to pretrain the near-miss words. In embedding spaces, different words that are semantically similar are likely to form semantic groups in which words with different properties are close together in distance. The continuous bag of words (CBOW) is a common model for word2vec [47]. The model is suitable for word embedding training in text datasets with fewer low-frequency words and more short sentences [48].

The main idea of the CBOW model is to use context words {*x*_1_,  *x*_2_, ..., *x*_*C*_} to predict the central word *W*_*i*_, where C is the window value (set to 5), *W*_*i*_ is the *i* word in word vector space, and {*x*_1_,  *x*_2_, ..., *x*_*C*_} is the one-hot coding (the corresponding index position of the word is 1, and the others are 0). The model calculation is divided into two processes: forward propagation and back propagation.

(1) Forward propagation.

Figure 4 shows the calculation process of forward propagation, where “氧气(oxygen)/乙炔(acetylene)/瓶 (bottle)/无 (no)/安全(safety)/距离(distance)” is taken as the dataset for illustration, and “bottle” is the predicted central word. Forward propagation is divided into two steps.

Step 1: Calculate the hidden layer *H*, which is a 1 × *N*-dimensional vector. *N* is the dimension of each word vector. The value is set to 100. The calculation formula is described as follows:
  (1) $$\begin{array}{c} H=\frac{1}{C}W_{0}\cdot \left(\sum_{i-1}^{C}x_{i}\right), \end{array}$$
where *W*_0_ is a *V* × *N*-dimensional matrix that connects the input vector and hidden layer, and *V* is the size of the word vector space. In the figure, the value is set to 6.
Step 2: Calculate the output vector *Y* of size 1 × *V*. *Y* (the word vector for “bottle” in this image) is a distributed representation of the predicted central word. To facilitate the calculation of errors during back propagation, the *softmax* function is used to normalize *H* × *W*_1_. The calculation formula is described as follows:
  (2) $$\begin{array}{c} Y=\text{softmax}\left(H\cdot W_{1}\right), \end{array}$$
where *W*_1_ is the weight matrix with a size of *N* × *V* to connect the hidden layer and the output layer.

*(2) Back Propagation*. The back propagation error is calculated according to *Y* of the center word and the one-hot encoding vector of this word. The values of *W*_0_ and *W*_1_ are continuously adjusted using the gradient descent method. During the training, each word is used as a central word; that is, *W*_0_ and *W*_1_ are modified *V* times. After the training, the one-hot coding vector of each word is computed in steps 1 and 2 and united with the trained *W*_0_ and *W*_1_ to accomplish the word vector of all words in the entire dataset.

#### 4.1.2. Convolution Layer

In the NLP domain, since the width of the convolution kernel is generally equal to the dimension *k* of the word embedding, the convolution kernel slides in only one dimension. We illustrate the process of convolution in Figure 4. In the example, the window value (the local word order length per convolution) *h* is set to 4. The process is divided into three steps. Step 1: the 4 × 4 matrix *X*_1:4_ corresponding to “氧气(oxygen)”/“乙炔(acetylene)”/“瓶(bottle)”/“无(no)” and convolution kernel *W* are substituted into formula 1 to obtain the feature mapping *C*_1_.

Step 2: due to the sliding step s=1, the window slides down one slot. We perform the same calculation by replacing *X*_1:4_ with *X*_2:5_ corresponding to “乙炔(acetylene)”/“瓶 (bottle)”/“无 (no)”/“安全 (safe).” Step 3: according to the first and second steps, an iterative operation is performed to obtain the feature mapping matrix *C*: 3 × 4. The calculation formula is described as follows:

(3) $$\begin{array}{c} c_{i}=f\left(w\cdot x_{i:i+h-1}+b\right), \end{array}$$

where *w* is the convolution kernel matrix representing the shared weight, and *x*_*i*:*i*+*h*−1_ is the connection matrix of the word embedding from the *i* word of a “description” or “location” to the *i*+*h* − 1 word. *b* is an offset term.  *f* is a nonlinear function, and in this study,  *f* is set to a rectified linear unit (ReLU).  Figure 5 shows the convolution process.

#### 4.1.3. Pooling Layer and Full Connection Layer

To represent richer features, the convolution kernel is set to different windows, and the same convolution kernel will run parallel operations [49]. Therefore, a sentence will generate feature vectors with different dimensions. The advantage of pooling is that it outputs a fixed-size matrix, reduces the dimensions of the output, and retains significant features with the maximum value *P*_*i*_(*i*=1,2,…, *m*). *P*_*i*_ is the maximum value of the vector by the i convolution operation, and m is the number of convolution kernels.

Dropout technology is adopted in the fully connected layer to prevent hidden layer neurons from self-adapting and to reduce overfitting [50]. The weight parameters of the fully connected layer are combined with *P*={*P*_1_, *P*_2_,…, *P*_*m*_} to calculate *Y*={*Y*_1_,…, *Y*_*t*_}. In this study, *t* is *t*_description_ (the number of “descriptions” tags) and *t*_*location*_ (the number of “locations” tags). After vector *Y* passes through the softmax layer, the probability distributions *L*={*L*_1_, *L*_2_,…, *L*_3_} of different labels are acquired by normalization calculations.  Figure 6 shows the process of pooling to the fully connected layer.

#### 4.1.4. Parameter Settings

According to the hyperparameter settings of CNN text classification in existing studies and through multiple comparison tests, the hyperparameters of this study are determined as shown in Table 3.

#### 4.1.5. Evaluation Metric

In this study, accuracy, recall, precision, and *F*_1_ score are used to evaluate the performance of the DL classification model. Formulas (4)–(7) define these metrics. Among them, recall can be understood as the ability to find crucial instances in the dataset, and precision represents the proportion of data points found by the model that is relevant to reality. The *F*_1_ score is a comprehensive evaluation of the model combined with recall and precision [51].

(4) $$\begin{array}{c} \text{accuracy}=\frac{\text{the number of correctly classified categories}}{\text{the sum of classified data}}\times 100\text{\%,} \end{array}$$

(5) $$\begin{array}{c} \text{precision}=\frac{TP}{TP+FP}, \end{array}$$

(6) $$\begin{array}{c} \text{recall}=\frac{TP}{TP+FN}, \end{array}$$

where *TP* is the number of positive samples predicted correctly, *FP* is the number of positive samples predicted incorrectly, and *FN* is the number of negative samples predicted incorrectly.

(7) $$\begin{array}{c} F_{1}\text{score}=\frac{2\times precision\times \text{Recall}}{\text{precision}+\text{Recall}}. \end{array}$$

### 4.2. Association Mining

This study utilizes the apriori association rule algorithm to analyze the associations between “type” and “location” classified by a CNN-based classifier. *D* is a set of all “types” and “locations.” If there is an association rule “location1 ⟶  type1” in which “location1” contains the “pipeline” item and “type1” contains the “electric shock” item, then there is a high probability of an electric shock accident occurring in the pipeline. “Location 1” and “type 1” (hereinafter abbreviated as *P*_1_ and *T*_1_) are both near-miss data item sets.

For association rule “*P*_1_⟶*T*_1_,” its support sup_(*P*__1__⟶*T*__1__)_ is used to measure the frequency of “*P*_1_⟶*T*_1_,” and the calculation formula is described as follows:

(8) $$\begin{array}{c} \sup_{\left(P_{1}⟶T_{1}\right)}=\frac{\text{count}\left(P_{1}\cap T_{1}\right)}{\text{count}\left(\text{D}\right)}, \end{array}$$

where count(*P*_1_∩*T*_1_) is the number of simultaneous transactions between *P*_1_ and *T*_1_, and count(D) is the total number of transactions.

Confidence conf_(*P*__1__⟶*T*__1__)_ measures the degree of credibility of “*P*_1_⟶*T*_1_”:

(9) $$\begin{array}{c} {\text{conf}}_{\left(P_{1}⟶T_{1}\right)}=\frac{\text{count}\left(P_{1}\cap T_{1}\right)}{\text{count}\left(P_{1}\right)}, \end{array}$$

where count(P_1_) is the number of transactions occurring in *P*_1_.

Rules whose support and confidence are both greater than a given threshold are called strong association rules [52].

In this study, the front and back items of association rules are “locations” and “types,” respectively, and each near-miss record is a single safety check record. The front and back items of association rules are limited. That is, there is only one item. Therefore, the algorithm can be improved to reduce the time cost of scanning by lowering the number of scans.

This algorithm can be divided into two steps as follows:

- Step 1: When finding the frequent 1-item set (the number of items contained in the frequent item set is 1), different from the traditional apriori algorithm, only the “location” item set is scanned instead of the item sets of “type” and “location” at the same time, thus saving scanning time. The corresponding support degree of each item is calculated, and an item set below the support threshold value is cut off to obtain a frequent 1-item set. The frequent 1-item set is connected with the “type” item set to obtain the candidate frequent 2-item set, and the candidate frequent 2-item set below the support degree is screened out to obtain the frequent 2-item set and its item statistics.
- Step 2: According to all frequent item sets mined in step 1, the confidence of each frequent item set is filtered whose value is greater than the small confidence; then, the frequent item set is a strong association rule.

This study explores what types of near misses may occur in a specific “location.” To show the relationship between them more intuitively, a network diagram is used to visualize them, as shown in Figure 7. The thickness of the line in the network represents the degree of correlation, and the size of the circle indicates the frequency of occurrence. The thickness is determined by the weight calculated from the support and confidence of the association rule. The weight is calculated in two steps: (1) normalizing “support” and “confidence” and (2) calculating the sum of the normalized “support” and “confidence” and then normalizing the result of the sum. The normalization can be calculated by formula (10). This solves the problem of inaccurate evaluation caused by different orders of magnitude of evaluation indexes. The statistical quantity of near-miss locations and near-miss types in hydropower projects is evenly distributed. If the support degree and confidence degree are set higher, some rules with strong practical relevance will be lost. In addition, the data in this study are large, so more valuable association rules can be obtained by setting these two values to smaller values. We set the support degree and confidence degree to be lower at 0.001 and 0.01, respectively.

(10) $$\begin{array}{c} y=\frac{x-x_{\min}}{x_{\max}-x_{\min}}, \end{array}$$

where *x* and *y* are the values before and after normalization, respectively, and *x*_max_ and *x*_min_ are the maximum and minimum values of the samples, respectively.

### 4.3. Sankey Diagram

The apriori algorithm can determine the strong association rule of “location ⟶ type” but cannot determine the distribution law of specific near-miss objects. The text corresponding to categories in strong association rules is processed by the Chinese word segmentation to obtain a more detailed near-miss distribution. For example, for “dam shoulder slot ⟶ fall from height,” (1) all descriptions of this association rule are collected as shown in Table 4, (2) the Jieba word segmentation package is used to segment the description in Chinese, and (3) words with large word frequency and significance as specific near-miss objects are selected to connect “location” and “type.” A Sankey diagram is drawn to describe the information flow of multiple strong association rules, in which the word frequency is used as the flow size.

## 5. Results and Discussion

### 5.1. CNN-Based Classification

To train the “location” and “type” classifiers with strong generalization ability, the dataset allocated according to section 3.4 is input into the constructed CNN DL text classification model. Furthermore, the model is evaluated by the accuracy, recall, precision, and F1 score.

The 8990 “description” data and the corresponding “location” data without labels generated in the Crane Beach Hydropower Station are taken to classify the “type” and “location,”, respectively, using the “type” classifier and the “location” classifier. The 8990 structured data are obtained for mining association rules “location ⟶ type.”

The average accuracy, average precision, average recall rate, and average F1 score rate of the “location” classifier were 90.19%, 81.90%, 84.43%, and 81.93%, respectively. The evaluation results of each category of the “location” classifier are shown in Figures 7 and8. The evaluation results of each category of the “type” classifier are shown in Table 5 and Figure 9.

In Figure 7, some categories are less effective, such as No. 28 “curtain” and No. 11 “drowning.” The similarity of drowning words is high, and the sample size is extremely small, which leads to a higher precision but lower recall. The sample size of the “curtain” is very small, leading to all evaluation metrics being 0. No. 1, No. 4, and No. 6 have higher recall but lower precision. This is because the texts tagged in these categories are similar to the texts tagged in other categories, and more other tags are classified as these.

In Table 5, “mechanical damage,” “collapse,” and “drowning” have higher precision but lower recall. The reason is that these categories have strong text features; thus, the classification precision is better, but the small sample size leads to a low recall.

Although precision, recall, and F_1_ scores indicate that the CNN performs better than other algorithms, they are unable to provide any information about how each category of “type” and “location” is misclassified. Thus, confusion matrices are introduced to focus on categories that are misclassified. In Figures 8 and 9, rectangles in the diagonal position represent the correct classification, while other rectangles represent the incorrect classification. Each row represents the actual category, and the column represents the predicted category.

As shown in Figure 8, since the descriptions of “No. 28” (“tunnel entrance”) and “No. 13“ (“inside tunnel”) are extremely similar, it is easiest to misclassify them. The top misclassified “type” shown in Figure 9 is “drowning.” The probability of “drowning” being misclassified as “civilized construction” (row 11, column 9) is 0.53. In the description of “civilized construction,” there is a large amount of “surface ponding.” Furthermore, the most striking feature that “drowning” describes is also “surface ponding,” so CNN classifiers easily confuse “drowning” with “civilized construction.” In addition, “collapse” has a 0.22 probability of being misclassified as “struck by objects” (row 8, column 10). After a collapse, there is a high probability of an object striking by accident. Therefore, the confusion between “collapse” and “struck by objects” can be explained by the symbiotic tendency. For a small number of categories that are easily confused, manual inspection is used for secondary classification to ensure classification accuracy.

### 5.2. Contrast Tests

Existing studies show that the short text classification effect of shallow machine learning is worse than that of DL [53]. Consequently, we do not consider shallow machine-learning algorithms and only compare four typical DL classification algorithms: recurrent neural network (RNN) [54], BERT [10], fast text [55], and long short-term memory (LSTM) [56].

Near-miss short texts on hydropower engineering construction have the characteristics of limited sentence length, compact structure, and independent expression, which make it possible for CNNs to handle such tasks [57]. Five DL classification algorithms classify the same dataset in the comparison test, and the same trained word embedding layer is used as the input layer.

As the number of categories classified in this study is too high to fully display the evaluation metrics of each category, the average value of each evaluation metric of the classifier is used for comparison with the CNN algorithm and other DL methods. As can be observed from Table 6, all metrics of the CNN algorithm are superior to those of other DL classification algorithms. Therefore, the CNN algorithm is adopted to classify the short text of near misses in hydropower engineering construction.

### 5.3. Association Rules

To acquire more objective association rules, labeled data are added to the association analysis dataset for more comprehensive data. Due to the large amount of data and the large number of label categories, the threshold of support and confidence were set at low levels of 0.02 and 0.20, respectively. A total of 31 strong association rules were mined. Some of the results are shown in Table 7.

To display more association information using a network diagram, we set the support degree and confidence degree lower at 0.001 and 0.01, respectively, and a total of 235 association rules are output. As shown in Figure 10, the larger circles of “civilized construction” and “struck by objects” indicate that these types of accidents are more likely to occur in the construction of hydropower engineering projects. According to the thickness of the line, “inside the tunnel” is prone to “collapse,” “vehicle injury,” “fire,” and other accident types, while “underground chambers” are prone to “fall from height,” “struck by objects,” “fire,” and other types of accidents.

Knowing which places are prone to accidents, safety managers can search for the corresponding original near-miss description data and perform a more in-depth and detailed analysis based on the specific association rules. For example, a tunnel is prone to collapse due to arch cracking, no anchor, nonstandard support, and so on. More valuable near-miss prevention objects can be learned by combining raw near-miss data with an association rule network.

Compared with the network diagram, the Sankey diagram displays more detailed and specific content and visually presents the frequency distribution and information flow of the specific near-miss objects, near-miss locations, and near types. We exhibit one of the Sankey diagrams in Figure 11 using 6 pairs of strong association rules. Some valuable hidden danger rules can be analyzed from the figure. For example, electric shock near misses are likely to appear in “dam shoulder slots” and “tailrace tunnels” due to the “inside of the distribution box.” Referring to the original text related to “inside the distribution box,” we can understand that “there is debris in the distribution box” is the cause of electric shock near misses, and it is more likely to appear in the “tailrace tunnel” and “dam shoulder slot.”

In addition, the “traffic ladder” of the “dam shoulder slot” has great potential to cause near misses of “falling from height.” Referring to the “traffic ladder” in the original text, we can find that the main reason for “fall from height” is that “there is no traffic ladder,” “the traffic ladder handrail is missing,” and “the traffic ladder has no protective railing.” Safety managers can quickly find the details of near misses and implement measures to prevent the emergence of these near misses through the Sankey diagrams combined with original text data.

## 6. Conclusion

The construction safety management of hydropower engineering is mainly based on the analysis of safety text data, but the recorded data are often inconsistent and messy data, so it is particularly difficult to directly obtain knowledge that can guide safety early warnings. In recent years, NLP technology combined with AI has provided the possibility for rapid and automatic analysis of text data in all walks of life.

To mine the valuable information hidden in the data of hydropower engineering construction near misses, this study developed a new model combining text classification and association mining. The purpose of text classification is to aggregate near misses in the same category and lay the foundation for subsequent data statistics. The association algorithm can be used to calculate the results of structured classification and find the association rules with strong practical significance.

To overcome the shortcoming that the association algorithm cannot analyze the near-miss description field that contains the most near-miss information, the method of word segmentation combined with the Sankey diagram was used to add abundant near-miss information to the association rules. Intuitive near-miss distribution visualization helps safety managers quickly find the causes of near misses and take measures to control them to reduce the possibility of accidents and improve the safety level of hydropower engineering construction sites. The model can mine massive texts and obtain more detailed rules and is also applicable to other fields of text mining.

Our research can better examine near-miss associations, but there are still some limitations. First, the work of making near-miss labels is completed by different people, which may lead to different classifications of the same near-miss types due to respective subjective opinions. Second, it is still necessary to manually check the near-miss classification results with poor performance in the classifier to ensure the accuracy of data involved in association rule mining. Third, the CNN-based model proposed was only used to evaluate the near-miss text dataset obtained from the Crane Beach Hydropower Station project. Future study is required to use unsupervised learning to improve the accuracy of near-miss data classification. In addition, the consistency of near-miss dataset classification models for different hydropower engineering projects can be further discussed.

## Figures and Tables

**Figure 1:** Data preparation process.

**Figure 2:** Text mining process of hydropower engineering construction near misses.

**Figure 3:** CNN classifier model framework.

**Figure 4:** CBOW forward propagation flowchart.

**Figure 5:** CNN convolution computation process.

**Figure 6:** Process of pooling to connection.

**Figure 7:** Precision, F_1_ score, and recall of “location” classification results.

**Figure 8:** Confusion matrix of “location” classification results.

**Figure 9:** Confusion matrix of “type” classification results.

**Figure 10:** “Location ⟶ type” network graph.

**Figure 11:** Sankey diagram of association rules.

**Table 1:** Portion of safety records for hydropower engineering projects.

检查日期 (check date)	隐患描述 (near-miss description)	隐患部位 (near-miss location)
2016/08/27	顶拱挂网施工, 汽车吊吊装范围未警戒防护 (roof arch hanging net construction, car hoisting range without warning protection)	引水上平施工支洞(12#∼13#之间)顶拱挂网施工, 汽车吊吊装范围未警戒防护 (construction of supporting tunnel (between #12 and #13) on the upper level of water diversion; construction of roof arch hanging net; no warning protection for the hoisting range of an automobile crane)
……		
2017/05/09	洞内照明设施不满足现场施工要求 (the lighting facilities in the cave do not meet the requirements of site construction)	左岸泵房交通洞 (left bank pump room traffic hole)

**Table 2:** Examples of near-miss label.

NO.	Near-miss description	“Type” label	Near-miss location	“Location” label
1	基础分局锚索施工排架二端过道未贴反光条提示过住车辆。(no reflective strip is attached to the second end corridor of the anchor cable construction rack in the basic subbureau.)	车辆伤害(vehicle injuries)	尾检北侧锚索施工排架 (construction of the anchor cable on the north side of the stern inspection)	排架 (bent)
2	现场电源线拆除后桩头裸漏 (after the removal of the power line on-site, the pile head is exposed to leakage.)	触电 (electric shock)	主变北侧交通洞洞口 (the main north side of the traffic hole)	洞口 (tunnel entrance)
3	一砂轮切割机无防护盖易造成操作人员伤害 (a grinding wheel cutting machine without a protective cover can easily cause injury to operators.)	机械伤害(mechanical injuries)	EL676马道 (EL676 berm)	马道 (berm)

**Table 3:** Setting of CNN model hyperparameters.

Embedding dimension	Filter size	Number of filters	Dropout probability	Learning rate
100	5	128	0.5	0.8

**Table 4:** Near-miss descriptions about “dam shoulder slot ⟶ fall from height.”

“Location”	Description	“Type”
Dam shoulder slot	坝肩槽EL635-EL625高程中间爬梯扶手焊点开裂2处, 存在安全隐患。(there are 2 cracked solder joints of the middle ladder handrail in the dam abutment grooves of EL635-EL625 that have safety risks.)	Fall from height
	临边防护及警示缺失。(lack of border protection and warning.)	
	…	
	坝肩槽EL74O通道端头未封闭开放, 存在坠落风险 (the end of the EL74°channel of the abutment groove is not closed and open, and there is a risk of falling.)	

**Table 5:** Precision, F1 score, and recall of “type” classification results.

No.	Label	Precision	Recall	*F*1 Score
1	Explosion	0.82	0.80	0.81
2	Vehicle injuries	0.72	0.66	0.69
3	Electric shock	0.97	0.95	0.96
4	Fall from height	0.82	0.87	0.85
5	Fire	0.89	0.77	0.82
6	Mechanical injuries	0.82	0.67	0.74
7	Lifting injuries	0.69	0.78	0.74
8	Collapse	0.86	0.58	0.69
9	Civilization construction	0.86	0.87	0.86
10	Object hit	0.71	0.79	0.75
11	Drowning	0.88	0.47	0.61
	Average	0.82	0.75	0.77

**Table 6:** Comparison of CNN classification algorithm and other deep learning methods.

Dataset	Classifier algorithm	Metrics			
		Accuracy	Precision	Recall	*F*_1_ score
*Near-miss type*	CNN	0.86	0.82	0.77	0.79
	RNN	0.85	0.79	0.74	0.76
	BERT	0.82	0.81	0.73	0.77
	Fast text	0.79	0.78	0.71	0.74
	LSTM	0.81	0.80	0.72	0.76

*Near-miss location*	CNN	0.90	0.82	0.84	0.83
	RNN	0.88	0.78	0.80	0.79
	BERT	0.85	0.75	0.78	0.76
	Fast text	0.81	0.73	0.75	0.74
	LSTM	0.86	0.77	0.78	0.77

**Table 7:** Results of association rule calculations.

No.	Location	Type	Support	Confidence
1	Gallery	Electric shock	0.02	0.36
2	Tailrace tunnel	Electric shock	0.13	0.33
3	Dam shoulder slot	Fall from height	0.03	0.30
4	Tunnel entrance	Civilization construction	0.05	0.29
5	Water inlet	Fall from height	0.05	0.29
6	Pipeline	Electric shock	0.06	0.28
7	Embankment slope	Struck by objects	0.03	0.28

## Data Availability

The data generated and analyzed during this research are available from the corresponding author by request.
